This article has been retracted.

# Bioheat transfer model of transcutaneous spinal cord stimulation-induced temperature changes

**DOI:** 10.7717/peerj.4921

**Published:** 2018-06-04

**Authors:** Luyao Chen, Ang Ke, Peng Zhang, Zhaolong Gao, Xuecheng Zou, Jiping He

**Affiliations:** 1 School of Optical and Electronic Information, Huazhong University of Science and Technology, Wuhan, China; 2 Neural Interface and Rehabilitation Technology Research Center, School of Automation, Huazhong University of Science and Technology, Wuhan, China; 3 Collaborative Innovation Center for Brain Science, Huazhong University of Science and Technology, Wuhan, China; 4 Advanced Innovation Center for Intelligent Robots and Systems, Beijing Institute of Technology, Beijing, China

**Keywords:** Transcutaneous spinal cord stimulation, Bioheat transfer, Finite element analysis, Temperature distribution

## Abstract

Transcutaneous spinal cord stimulation (tSCS) has been extensively studied due to its promising application in motor function restoration. Many previous studies have explored both the essential mechanism of action and the methods for determining optimal stimulation parameters. In contrast, the bioheat transfer analysis of tSCS therapy has not been investigated to the same extent, despite widely existing, and being of great significance in assuring a stable and thermally safe treatment. In this paper, we concentrated on the thermal effects of tSCS using a finite element-based method. By coupling the electric field and bioheat field, systematic finite element simulations were performed on a human spinal cord model to survey the influence of anatomical structures, blood perfusion, and stimulation parameters on temperature changes for the first time. The results show that tSCS-induced temperature rise mainly occurs in the skin and fat layers and varies due to individual differences. The current density distribution along with the interactions of multiple biothermal effects synthetically determines the thermal status of the whole spinal cord model. Smaller stimulation electrodes have a higher risk of thermal damage when compared with larger electrodes. Increasing the stimulation intensity will result in more joule heat accumulation, hence an increase in the temperature. Among all configurations in this study that simulated the clinical tSCS protocols, the temperature rise could reach up to 9.4 °C on the skin surface depending on the stimulation parameters and tissue blood perfusion.

## Introduction

Transcutaneous spinal cord stimulation (tSCS) is a non-invasive and low-cost technique that has already shown promising effects in the neuromodulation of motor control (Gerasimenko et al., 2015a, 2015b; Krenn et al., 2015; Minassian et al., 2016). By passing currents through the skin and targeting neural circuits in the lumbosacral spinal cord, lower limb motor function could be restored to a certain extent for patients with spinal cord injury. Despite the breakthroughs in both modeling studies and clinical experiments, the risk of thermal damage caused by tSCS cannot be ignored. Skin burns have been suggested to be the major obstacle for transcutaneous electrical stimulation-based therapies according to Nadler’s retrospective questionnaire study (Nadler et al., 2003). Thermal damage caused by continuous stimulation induced an uncomfortable sensation, thus restricting the further application of the non-invasive therapy (Patriciu et al., 2001, 2005; Lagopoulos & Degabriele, 2008). Previous reports on the skin burns caused by transcutaneous electrical stimulation indicated the significant role of the electrode properties and stimulation parameters on the bioheat accumulation and transference (Balmaseda et al., 1987; Patriciu et al., 2001; Ford et al., 2005; Satter, 2008; Sharma et al., 2011).

Commonly, joule heat will be generated in any electrical field where electrical current is circulating. Thus, it is inevitable that thermal energy is accumulating during tSCS as the electrical current is delivered through the biological tissues by the electrode pairs. Additionally, the Pennes model (Pennes, 1948) indicated that the contribution of physiological procedures, such as the metabolic heat generation and blood perfusion, in determining the thermal status. The synthetic and complex interaction of these internal and external heat sources and heat sinks could result in either slight or severe temperature rises during electrical stimulation treatments depending on the tissue properties and stimulation parameters.

Finite element calculation is an efficient tool to explore both the electrical and thermal field distribution with the help of accurate anatomical models. Previous numerical studies based on spinal cord modeling have already clarified valuable information regarding the electrical field distribution and nerve fiber response. It was demonstrated that both the anterior and posterior root fibers can be activated by tSCS, which covers the targeting regions of epidural spinal cord stimulation, and offers evidence for the lower limb muscle responses induced by transcutaneous posterior root stimulation (Ladenbauer et al., 2010). More recently, Kuck’s group concluded from their spinal cord and axon modeling study that the current density induced by tSCS is sufficiently strong to evoke functional modulation (Kuck, Stegeman & van Asseldonk, 2017). Those studies showed that tSCS with proper stimulation parameters can become a promising noninvasive modality in the rehabilitation of people suffering related neural disorders. While most of the existing research focuses on verifying the efficacy and searching for a proper stimulation protocol for tSCS (Ladenbauer et al., 2010; Danner et al., 2011; Gerasimenko et al., 2015a), insufficient efforts have been put towards investigating the bioheat transference of this promising therapy which is significant in evaluating the safety of the treatment.

In this paper, we tested the impact of several biological and stimulation properties on the bioheat transfer, including the thicknesses of the skin and fat layers, the blood perfusion rate of the dermis and neural tissue, electrical stimulation intensities, and the size of the stimulation electrode. A finite element human spinal cord model was built to simulate the electrical and thermal field during continuous tSCS. Parameter sweeping studies were used to compare the electrical field distribution and the temperature changes during stimulation. Prior to clinical research, this work provides a systematic description of analyzing the thermal issues related to the tSCS treatment.

## Materials and Methods

### Finite element spinal cord model with transcutaneous electrodes

A three-dimensional human spinal cord model was constructed based on a model from a previous study (Ladenbauer et al., 2010). We first constructed a two-dimensional model including tissues such as the gray matter (GM), white matter (WM), cerebral spinal fluid (CSF), epidural fat (EF), vertebrae (Vert), and muscles, by referring to the geometry and size of Ladenbauer’s model. The model was then imported to COMSOL Multiphysics (COMSOL Inc., Burlington, MA, USA), and layered cylinders were used to represent the boundary of the fat and three-layered skin with stratum corneum (SC), epidermis (ED), and dermis. A symmetrical three-dimensional model was finalized by extruding the surface model as shown in Fig. 1A. In this work, to study the impact of individual anatomical differences on temperature variance, different models with various skin and fat layer thicknesses were formulated and simulated. It is believed that the thickness of the surface skin layers outside the dermis is approximately 100 μm and that of the SC layer varies from 10 to 40 μm. In the simulations, SC thicknesses of 10, 20, 30, and 40 μm were tested, and the corresponding ED layer was 90, 80, 70, or 60 μm in thickness, respectively. Furthermore, previous studies set the thickness of the fat layer at 10 mm (Lv & Liu, 2007) or 4.4 mm (Xu et al., 2008) and thickness of the dermis layer at 1.5 mm (Xu et al., 2008) or 2 mm (Lv & Liu, 2007). Therefore, we created models with dermis thicknesses of 1, 1.5, and 2 mm, and models with fat thicknesses from 4 to 16 mm with 2 mm steps to cover the reference range. As the control model, the thicknesses of the SC/ED/dermis/fat were set to 20/80 μm/2/10 mm, respectively. Before tSCS, the 1 × 1 cm × 2 mm (length × width × depth) stimulation electrode was symmetrically placed over the spine and a 5 × 5 cm × 2 mm (length × width × depth) return electrode was fixed over the abdomen of the model as shown in Figs. 1B and 1C, respectively. In this work, stimulation electrodes with the side lengths of 1, 1.5, and 2 cm were made to simulate the impact of electrode size on the thermal accumulation during tSCS.

**Figure 1:** Human spinal cord model and the transcutaneous electrodes. (A) Two-dimensional spinal cord model and the extruding direction to form the three-dimensional model. (B) The three-dimensional full spinal cord model with the stimulation electrode placed on the surface of the skin. The side length of the electrode is 1 cm. The surface highlighted in blue color is defined as the stimulation surface. (C) The spinal cord model with the return electrode. The side length of the return electrode is 5 cm. The surface highlighted in blue color is defined as the return surface. (D) The central cross-sectional surface of the spinal cord model across the centers of the stimulation surface and the return surface. (E) Detailed view of the cross-sectional surface of the spinal cord. A central line across the center of the stimulation surface and the return surface is defined in red. (F) Magnified view of the central parts of the spinal cord.

Before starting the simulations, the spinal cord model with electrodes was meshed using tetrahedral and swept methods. The main element size parameters used to define the mesh settings included the maximum element size, minimum element size, maximum element growth rate, curvature factor, and resolution of narrow regions. We first used a free tetrahedral mesh for the stimulation and return electrodes with element size parameters of 0.0219, 0.0016 m, 1.4, 0.4, and 0.7 corresponding to the above-mentioned parameters, respectively. Since the structure of the SC and ED layers are characterized by an extremely high surface area-to-thickness ratio, a prior triangular mesh with element size parameters of 0.005, 2.67E-4 m, 1.08, 0.3, and 0.95 was applied to the skin surfaces followed with a swept mesh for the whole volumes of the two tissue types. The distribution properties of the swept mesh were set as a fixed number of elements, four for the SC layer and 16 for the ED for the control model, and varied correspondingly with the thickness of the skin layers. A finer mesh was chosen for the skin layers, while a coarser mesh was applied to the remaining tissues using a free tetrahedral method. The corresponding element size parameters were 0.0319, 0.00399 m, 1.45, 0.5, and 0.6 respectively. The mesh statistics of the control model are shown in Table 1. A convergence study was conducted to determine the proper meshing sizes by tracking the peak temperature with the total meshing elements. Consequently, a trade-off between the computational time and accuracy was reached at a total of 0.63 million elements as shown in Table 1. In order to illustrate and analyze the simulation results, two reference surfaces and a reference line of the spinal cord model were defined, i.e., the skin surface beneath the stimulation electrode as shown in Fig. 1B, the cross-sectional surface as shown in Fig. 1D, and the red line as shown in Fig. 1E. Figure 1F shows the detailed anatomical structure of the spinal cord.

**Table 1:** The mesh statistics.

Mesh statistics parameter	Value
Number of tetrahedral elements	3.1E5
Number of prism elements	3.2E5
Number of triangular elements	1.0E5
Number of Quadrilateral elements	1.2E4
Minimum element quality	0.7818
Average element quality	0.03521
Element volume ratio	9.67E-7
Element volume	0.01157 m^3^

**Note:**

The stimulation electrode size is 1cm in length and width, the thickness of the tissues are: fat = 10 mm, dermis = 2 mm, epidermis = 80 μm, SC = 20 μm.

### Bioheat model during tSCS

During tSCS, the heat sources include joule heat and metabolic heat, while the heat dissipation process consists of the blood perfusion effect and heat convection effect between air and skin or electrode surface as shown in Fig. 2. Based on the Pennes model (Pennes, 1948), we added the joule heat induced by the electrical field as an extra heat source as expressed in Eq. (1). Furthermore, the heat convection is considered in the SC and electrode surfaces as shown in the last term of the Eq. (1).

**Figure 2:** Bioheat transfer model during tSCS.

(1) $$c\rho {{\partial T} \over {\partial t}} = \nabla \cdot \left( {k\nabla T} \right) + {\left| {\vec J} \right|^2}/\sigma + {Q_{\rm{M}}} - {\omega _{\rm{b}}}{\rho _{\rm{b}}}{c_{\rm{b}}}\left( {{T_{\rm{b}}} - T} \right) - h\left( {T - {T_{{\rm{ext}}}}} \right) $$

Where *T*, *c*, and *ρ* represent the temperature (°C), specific heat (J/kg-K), and density (kg/m^3^) of a specific tissue type, respectively, and *T*_b_, *c*_b_, *ρ*_b_, and ω_b_ represent the blood temperature (°C), blood specific heat (J/kg-K), blood density (kg/m^3^), and blood perfusion rate (s^−1^), respectively, *k* is the thermal conductivity (W/m-K), *t* represents stimulation time (s), *J* represents the current density distribution (A/m^2^), σ is the electric conductivity (S), *Q*_M_ is the metabolic heat (W/m^3^), *h* is convective heat transfer coefficient (W/m^2^-K), and *T*_ext_ is the external air temperature (°C). Specifically, the initial temperature of the biological tissues were set at 37 °C, *T*_ext_ at 25 °C, and *h* is 1.86 and 7.9 for the skin surface (de Dear et al., 1997) and electrode surface (The Engineering ToolBox, 2018), respectively. In the steady state, the Laplace equation, ∇·(σ∇*V*) = 0, is used to determine the potential distribution *V* (V) among the tissues, which could then be used to calculate the electric field and current density in a further step. The initial electric condition was determined by *V* = 0. Note that the outer boundaries of the spinal cord were selected as electrical insulations, where ∂*V*/∂*n* = 0. Except for the skin surface, which was treated as a heat convective flux, other outer boundaries were thermally insulated and defined as ∂*T*/∂*n* = 0. All the internal boundaries with two interfacing tissue layers were treated as electrically and thermally continuous. Additionally, in this work, we treat metabolic heat generation as zero or constant values, as listed in Table 2.

**Table 2:** Properties of the biological tissues.

Biological tissues	Blood perfusion rate ω (1/s)	Metabolic heat generation *Q_M_* (*W/m*^3^)	Thermal conductivity *k* (*W/m-K*)	Electrical conductivity σ (S/m)
SC	0	368.1	0.235	0.0025
ED	0	368.1	0.235	0.15
Dermis	0.012	368.1	0.445	1.62
Fat	0.0035	368.3	0.185	0.02383
Abdomen	0.3	180	0.52	0.0414
Muscle	0.00017	690	0.498	0.08^1^/0.5^2^
Vert	0.0003	368.3	0.3	0.0285
EF	0.0035	368.3	0.21	0.04
CSF	0	0	1.12	1.7
GM	0.012	10,000	0.565	0.23
WM	0.012	10,000	0.503	0.083^1^/0.6^2^

**Notes:**

1 Transversal;

2 Longitudinal.

Schwan & Kay (1957), Tavernier, Dierickx & Hinsenkamp (1992), Gabriel, Gabriel & Corthout (1996), Xu et al. (2008), Smith & Zhu (2010), Danner et al. (2011), Parazzini et al. (2014), and Miller et al. (2016).

In the present simulation studies, except for the isotropic electrical properties of the muscles and WM, all biological compartments are considered as pure resistors under constant stimulation. The electrical and thermal properties of the tissues are listed in Table 2. As for the stimulation intensity, we modeled the commonly used alternating current input as an equivalent constant value under the principle that the total joule heat energy caused by both stimulation signals during the same amount of stimulation period are the same. Thus, a sequence of biphasic pulses repeated at *f*_L_ with an amplitude of *I_p_* would be equivalent to a constant current *I*_rms_ as represented in Eq. (2), where *N* indicates the number of the pules at a frequency of *f*_H_.

(2) $${I_{{\rm{rms}}}} = {I_p}{\rm{*}}\sqrt {N{\rm{*}}{f_{\rm{L}}}/{f_{\rm{H}}}} $$

To cover most of the parameter settings utilized in recent clinical applications, we swept the constant current from 0 to 40 mA in this work. The total stimulation time was set at 15 min, which was enough for the model to reach a stable peak temperature (Chen et al., 2017; Khadka et al., 2017). The time-dependent study was chosen with a maximum time step of 10 s under a peak relative tolerance of 0.01. A parametric sweep was added to test the impact on the biothermal status of the blood perfusion rate and stimulation intensity on the control model as described in “Finite Element Spinal Cord Model with Transcutaneous Electrodes.” The sweeping parameters were 0, 5, 10, 20, 30, and 40 mA for the stimulation intensity, 0, 0.025, 0.05, and 0.1 s^−1^ for the blood perfusion rate of the dermis, and 0, 0.004, 0.008, and 0.012 s^−1^ for the blood perfusion rate of the WM/GM. Simulations aimed at testing the impact of the anatomical parameters set the stimulation intensity and the blood perfusion rate of the dermis and WM/GM at 20 mA, 0.025, and 0.012 s^−1^, respectively. As for data analysis, temperature change curves vs. stimulation time were recorded, as well as the electrical and thermal distributions among the reference faces or line induced by the various tSCS configurations.

## Results

### Effects of skin or fat thickness on the temperature distribution induced by tSCS

The thicknesses of the skin and fat layers vary by individual (Mathias & Srinivas Murthy, 2017). Figures 3A–3D, 3E–3H, and 3I–3L show the results of different SC/ED thicknesses, dermis thicknesses, and fat thicknesses, respectively, on the temperature distribution during tSCS at 20 mA. Peak temperatures for the skin layers, fat, abdomen, muscles, and the Vert at the end of the stimulation varied with the changes of tissue thickness, whereas those of the EF, CSF, and WM/GM remained the same. Figures 3B, 3F, and 3J show the temperature distribution along the reference line defined in Fig. 1E. The results show that with an increase in the SC layer thickness or decrease in the dermis layer thickness, the temperature of the skin and fat layers becomes higher, which is consistent with the results shown in Figs. 3A and 3E. The peak temperature of the whole biological model reached as high as 40.8 and 40.0 °C when the thicknesses of SC/ED/dermis were 40/60 μm/2 mm and 20/80 μm/1 mm, respectively. As for the changes of the fat thickness, no consistent pattern could be identified for the peak temperature of the skin and fat layers from Figs. 3I–3J. In contrast, the peak temperatures of the abdomen, muscles, and Vert decreased with an increase in the fat thickness to 12 mm. However, for even thicker fat, the peak values remained unchanged. We recorded the coordinates of the points with the peak temperature for each tissue type and tracked their temperature change curves over time as shown in Figs. 3C–3D, 3G–3H, and 3K–3L for different variables. A pattern seen across the figures, is that the temperature of the skin and fat layers rises rapidly once the stimulation is turned on and then reaches a plateau. The SC and ED layers share similar temperature distribution and the rising curves of the peak temperature points almost overlapped in every simulation. With the decrease of the SC layer thickness and increase of the dermis layer thickness, the peak temperature points of the dermis layer were closer to those of the SC/ED layers as shown in Figs. 3C and 3G. Similarly, the rising curves of the peak temperature points in the muscles and Vert overlapped in each of the simulations and that of the EF, CSF, and GM/WM overlapped in all simulations. The results revealed the significance of designing customized stimulation protocols for individuals by considering the thicknesses of the skin and fat layers.

**Figure 3:** Effects of the tissue thickness on the thermal status during tSCS. (A–D) The thickness of the SC layer varies from 10 to 40 μm. Dermis = 2 mm. Fat = 10 mm. (E–H) The thickness of the dermis layer varies from 1 to 2 mm. SC = 20 μm. Fat = 10 mm. (I–L) The thickness of the fat layer varies from 4 to 16 mm. SC = 20 μm. Dermis = 2 mm. (A), (E), (I) The peak temperature values of each tissue type at the end of tSCS. (B), (F), (J) Temperature distribution at the end of tSCS along the reference line defined in Fig. 1E. Insets in (B) and (F): Magnified view of the parts across the SC/EF/Dermis skin layers. (C–D), (G–H), (K–L) Temperature rising curves of the points with peak temperature variance for each tissue type. The stimulation intensity is 20 mA, the stimulation electrode side length is 1 cm, and the blood perfusion rate of the dermis and WM/GM are 0.025 and 0.012 s^−1^, respectively.

### Effects of blood perfusion on the temperature distribution induced by tSCS

It is known that blood perfusion varies with tissue temperature (Tompkinsn et al., 1994); whether and to what extent the varied blood perfusion rate could influence bioheat transfer and the biothermal status will be investigated in this section. In this section, the stimulation intensity was chosen to be 20 mA and the electrode was 1 cm in side length. Figures 4A–4B and 5A–5B show the peak temperature values of each tissue type and temperature distribution along the reference line when the tSCS finished. The results suggest that temperature changes induced by tSCS with different blood perfusion rate mainly occur in the skin and fat layers, abdomen, muscles and Vert, for the dermis, and in the Vert, EF, CSF, and WM/GM for the WM/GM.

**Figure 4:** Effects of the blood perfusion of the dermis layer on the thermal status during tSCS. (A) The peak temperature values of each tissue type at the end of the electrical stimulation. (B) Temperature distribution along the reference line at the end of tSCS. (C–D) Temperature rising curves of the points with peak temperature variance for each tissue type. The stimulation intensity is 20 mA, the stimulation electrode side length is 1 cm, and the blood perfusion rate of the WM/GM is 0.012 s^−1^. The unit of the blood perfusion rate is s^−1^.

**Figure 5:** Effects of the blood perfusion of the WM/GM on the thermal status during tSCS. (A) The peak temperature of each tissue type at the end of the electrical stimulation. (B) Temperature distribution along the reference line at the end of tSCS. (C) Temperature rising curves of the points with peak temperature variance for the spine tissues. The stimulation intensity is 20 mA, the stimulation electrode side length is 1 cm, and the blood perfusion rate of the dermis layer is 0.025 s^−1^. The unit of the blood perfusion rate is s^−1^.

The peak temperature of the whole biological model could reach 41.7 °C if the blood perfusion rate of the dermis layer was set to 0. Figures 4C and 4D shows the peak temperature rising curves of the biological tissues at the end of the stimulation. In general, the peak temperature decreases with an increasing blood perfusion rate of the dermis, consistent with previous publications (Elwassif et al., 2006; Xu et al., 2008). Specifically, the peak temperature of the whole model is 41.7, 38.8, 38.3, and 37.9 °C when the dermis blood perfusion rate is 0, 0.025, 0.5, and 0.1 s^−1^, respectively. The temperature distribution among the reference surfaces in Fig. 6 demonstrates the influence of the dermis blood perfusion on the thermal status after 15 min tSCS. The peak temperature of the whole model is always located in the SC skin layer and the ED layer has a similar temperature distribution to the SC layer. With a decrease in the dermis blood perfusion, the difference of the peak temperature between the dermis and SC/ED becomes smaller. Moreover, with lower blood perfusion rates, heat seems more likely to accumulate in the deeper tissues, which may cause risk to the deep tissues, if intense stimulation parameters are applied at the same time.

**Figure 6:** Temperature distribution at the end of stimulation for varied blood perfusion rate of the dermis layer. (A–C) The blood perfusion rate of the dermis is 0 s^−1^. (D–F) The blood perfusion rate of the dermis is 0.025 s^−1^. (G–I) The blood perfusion rate of the dermis is 0.05 s^−1^. (J–L) The blood perfusion rate of the dermis is 0.1 s^−1^. (A, D, G, J) The temperature distribution on the cross-sectional surface for different perfusion rate of the dermis layer. (B, E, H, K) The magnified view of the hot area, i.e. the skin and fat layers (circled in (A, D, G, J) respectively). (C, F, I, L) The temperature distribution of the abdomen, muscles and the vertebrae. The stimulation intensity is 20 mA, the stimulation electrode side length is 1 cm, and the blood perfusion rate of the WM/GM is 0.012 s^−1^. The maximum and minimum temperature values are shown with the corresponding color bars in each panel. Unit: °C.

Similarly, temperature rising curves of the points with peak temperature variance for the spine tissues are shown in Fig. 5C and the temperature distribution in the spine are shown in Fig. 7 with different blood perfusion rate of the WM/GM. The temperature variance of the neural tissues is about 0.2 °C for 0.012 s^−1^. However, without blood perfusion of the WM/GM, the peak temperature of the tissues in the spine, which is always located in the WM/GM, would be 37.4 °C. This may due to the fact that slower blood perfusion in the WM/GM results in greater heat accumulates in the matters according to the bioheat model in Eq. (1). The extra heat dissipates from the deep neural tissues to the surrounding CSF, EF, and Vert, resulting in temperature rises in these tissues.

**Figure 7:** Temperature distribution of the spine at the end of stimulation for varied blood perfusion rate of the WM/GM. (A) The blood perfusion rate of the GM/WM is 0 s^−1^. (B) The blood perfusion rate of the GM/WM is 0.004 s^−1^. (C) The blood perfusion rate of the GM/WM is 0.008 s^−1^. (D) The blood perfusion rate of the GM/WM is 0.012 s^−1^. Tissues include vertebrae, epidural fat, CSF, WM, and GM. The stimulation intensity is 20 mA, the stimulation electrode side length is 1 cm, and the blood perfusion rate of the dermis is 0.025 s^−1^. The maximum and minimum temperature values are shown with the corresponding color bars in each panel. Unit: °C.

### Effects of the electrode size on the temperature distribution induced by tSCS

Setting the stimulation intensity at 40 mA, three models, with stimulation electrode with a side length of 1, 1.5, or 2.0 cm, were simulated to investigate the effects of electrode size on the temperature distribution during tSCS.

Theoretically, a larger contact area means smaller current density, thus less joule heat is produced. Hence, larger-size electrodes should cause smaller temperature rises. Figure 8 shows the current density distribution of the cross-sectional and stimulation surfaces. The middle three figures magnify the regions near the stimulation electrode and show relatively higher current density distribution than the deep tissues. The peak current density of the stimulation surface using 1-cm electrode is 1.66 and 2.52 times of that using the 1.5 and 2-cm electrode, respectively. Due to the edge effect, tissues beneath the edges of the stimulation electrode especially attract more current density. As for the thermal field, Fig. 9A shows the peak temperature of the biological tissues and Fig. 9B shows the temperature distribution along the reference line using electrodes with different sizes. Accordingly, temperature variance between the three electrodes mainly occurred in the skin layers and fat layer. As for the abdomen, muscles, and Vert, the peak temperature variance was relatively small and less than 0.3 °C. With the increase of the electrode size, the peak temperature rise of the whole model caused by tSCS decreased from 9.4 °C for the 1-cm electrode to 2.1 °C for the 1.5-cm electrode, and becomes negligible when the side length is increased to 2 cm. For a detailed view, Fig. 10 shows the temperature distribution across the cross-sectional surface and the stimulation surface at the end of the stimulation. To exaggerate the temperature differences induced by the electrode sizes, we magnified the specific parts circled in the first row and separately demonstrated the temperature distribution in the abdomen, muscles, and Vert as shown in the second and third row. The results indicate that larger electrodes deliver weaker current density and cause smaller temperature rises, which is consistent with the theory. It can be concluded that larger stimulation electrodes are thermally safer for tSCS and could bear more intense stimulation when compared with smaller ones.

**Figure 8:** Current density distribution of the reference surfaces for stimulation electrodes with different sizes. (A–C) The side length of the stimulation electrode is 1 cm. (D–F) The side length of the stimulation electrode is 1.5 cm. (G–I) The side length of the stimulation electrode is 2 cm. (A, D, G) The current density distributions on the cross-sectional surface for different electrode sizes. (B, E, H) The magnified view of the circled area in (A, D, G) respectively, i.e. the skin and fat layers. (C, F, I) The current density distributions on the stimulation surface. The stimulation intensity is 40 mA, and the blood perfusion rate of the dermis and WM/GM are 0.025 s^−1^ and 0.012 s^−1^ respectively. The maximum and minimum temperature values are shown with the corresponding color bars in each panel. Unit: A/m^2^.

**Figure 9:** Effects of the stimulation electrode size on the thermal status during tSCS. (A) The peak temperature values of each tissue type at the end of the electrical stimulation with different electrode sizes. (B) Temperature distribution along the reference line at the end of tSCS. The stimulation intensity is 40 mA, and the blood perfusion rate of the dermis and WM/GM are 0.025 and 0.012 s^−1^, respectively.

**Figure 10:** Temperature distribution induced by tSCS using electrodes with different sizes. (A–D) Electrode side length = 1 cm. (E–H) Electrode side length = 1.5 cm. (I–L) Electrode side length = 2 cm. (A, E, I) The temperature distributions on the cross-sectional surface for different electrode sizes. (B, F, J) The magnified view of the hot area (circled in (A, E, I) respectively), i.e. the skin and fat layers. (C, G, K) The temperature distribution of the abdomen, muscles and the vertebrae. (D, H, L)The temperature distribution on the stimulation surface. The stimulation intensity is 40 mA, and the blood perfusion rate of the dermis and WM/GM are 0.025 s^−1^ and 0.012 s^−1^ respectively. The maximum and minimum temperature values are shown with the corresponding color bars in each panel. Unit: °C.

### Effects of stimulation intensity on the temperature distribution induced by tSCS

Unlike ESCS where the stimulation electrode is placed very close to the modulating targets, tSCS uses electrodes on the skin surface. Consequently, to activate the nerves or neurons locate in the WM/GM, more amount of electric power is needed to be delivered through the layered tissues. According to Eq. (1), the input current intensity directly affects the amount of joule heat accumulation in a square way, therefore negligible temperature rises may occur with an increase of the input current. To verify the effects of stimulation intensity on temperature variance, we swept the equivalent input current from 5 to 40 mA, covering a wide range of stimulation signals with different pulse widths, repeated frequencies, and amplitudes used in recent clinical applications (Gerasimenko et al., 2015a, 2015b; Krenn et al., 2015; Minassian et al., 2016), according to Eq. (2). In addition, a simulation with stimulation intensity at 0 mA was added to show the thermal status without tSCS. It indicates that the current density increases with the increasing stimulation intensity as shown in the overview of the cross-sectional surface and magnification of the layers with high current density in Fig. 11. The current density was mainly delivered through layers of tissues into the targeted spine, and increased as shown in the third row of Figs. 11A–11F. The shunting effect due to the larger electrical conductivity of the CSF compared with the WM/GM was also verified as larger current density distributed more among the CSF than the deep neural tissues.

**Figure 11:** Current density distribution for different stimulation intensities. (A–C) Stimulation time = 0 mA. (D–F) Stimulation time = 5 mA. (G–I) Stimulation time = 10 mA. (J–L) Stimulation time = 20 mA. (M–O) Stimulation time = 30 mA. (P–R) Stimulation time = 40 mA. (A, D, G, J, M, P) The current density distribution on the cross-sectional surface for different stimulation intensities. (B, E, H, K, N, Q) the middle one is magnified detailed view of the circled area in (A, D, G, J, M, P) respectively, i.e. the skin and fat layers. (C, F, I, L, O, R) The temperature distribution of the vertebrae, epidural fat, CSF, WM, and GM. The stimulation electrode side length is 1 cm, and the blood perfusion rate of the dermis and WM/GM are 0.025 s^−1^ and 0.012 s^−1^ respectively. The maximum and minimum current density values are shown with the corresponding color bars in each panel. Unit: A/m^2^.

The peak temperature of each tissue type, temperature distribution along the reference line, and temperature change curves of points with peak temperature variance induced by different stimulation intensities are shown in Fig. 12. Generally, temperature variance between the groups with different stimulation intensities mainly occurred in all tissues except the CSF and WM/GM. Input signals with an equivalent current less than 20 mA are thermally safe for tSCS therapy. Temperature rise could be as high as 5 and 9.4 °C at 30 and 40 mA, respectively. Figure 11E indicates that the peak temperature of the SC increases rapidly, reaches its peak value in 340, 320, and 250 s for 20, 30, and 40 mA, respectively, and then plateaus. In comparison, the final temperature in the skin and fat layers are lower than the initial temperature at 0 and 5 mA, and very close to 37 °C at 10 mA. This may due to the fact that the weak stimulation current-induced heat accumulation is relatively small, while the heat convection effect of the skin surface dissipates the heat away, lowering the temperature of the skin and fat layers. The synthetic interaction of the heat sources and heat sinks at stimulation intensities lower than 10 mA causes the rising curves to be different from those at higher stimulation intensities, as shown in Fig. 12E. Detailed temperature distribution among the reference surfaces and the spine are shown in Figs. 13 and 14. In cases of stimulation under 10 mA, the temperature distributions are similar and the peak temperature rise of the whole model is no more than 0.2 °C. However, if the stimulation intensity is set to be more than 20 mA, the temperature of the tissues except the EF, CSF, and WM/GM rise and will increase with the stimulation intensity as shown in Fig. 14. Skin can be thermally damaged by a persistent heating above the safe limit, i.e., 45 °C (Moritz & Henriques, 1947; Pearce et al., 1983; Prausnitz, 1996) or 44 °C (Jiang et al., 2002). According to the assumptions of Henriques and Moritz (Henriques, 1947; Jiang et al., 2002), the extent of tissue thermal damage is dependent not only on the temperature but the exposure time and the properties of the tissues, such as frequency factor and activation energy. Hence, the extra multiple factors are essential to be considered for a more accurate safe threshold calculation in future work.

**Figure 12:** Effects of the stimulation intensity on the thermal status during tSCS. (A) The peak temperature of each tissue type at the end of the electrical stimulation with different stimulation intensities. (B) Temperature distribution along the reference line at the end of tSCS. (C–D) Temperature rising curves of the points with peak temperature variance for each tissue type for stimulation intensity of 20, 30, and 40 mA. (E) Temperature rising curves of the points with peak temperature variance for each tissue type for stimulation intensity of 0, 5, and 10 mA. The stimulation electrode side length is 1 cm, and the blood perfusion rate of the dermis and WM/GM are 0.025 and 0.012 s^−1^, respectively.

**Figure 13:** Temperature distribution at the end of stimulation for varied stimulation intensity from 0 mA to 10 mA. (A–D) The stimulation intensity is 0 mA. (E–H) The stimulation intensity is 5 mA. (I–L) The stimulation intensity is 10 mA. (A, E, I) The temperature distributions on the cross-sectional surface for different stimulation intensities. (B, F, J) The magnified view of the hot area (circled in (A, E, I) respectively), i.e. the skin and fat layers. (C, G, K) The temperature distribution of the abdomen, muscles and the vertebrae. (D, H, L) Shows temperature distribution of the vertebrae, epidural fat, CSF, WM, and GM. The stimulation electrode side length is 1 cm, and the blood perfusion rate of the dermis and WM/GM are 0.025 s^−1^ and 0.012 s^−1^ respectively. The maximum and minimum temperature values are shown with the corresponding color bars in each panel. Unit: °C.

**Figure 14:** Temperature distribution at the end of stimulation for varied stimulation intensity from 20 mA to 40 mA. (A–D) The stimulation intensity is 20 mA. (E–H) The stimulation intensity is 30 mA. (I–L) The stimulation intensity is 40 mA. (A, E, I) The temperature distributions on the cross-sectional surface for different stimulation intensities. (B, F, J) The magnified view of the hot area (circled in (A, E, I) respectively), i.e. the skin and fat layers. (C, G, K) The temperature distribution of the abdomen, muscles and the vertebrae. (D, H, L) Shows temperature distribution of the vertebrae, epidural fat, CSF, WM, and GM. The stimulation electrode side length is 1 cm, and the blood perfusion rate of the dermis and WM/GM are 0.025 s^−1^ and 0.012 s^−1^ respectively. The maximum and minimum temperature values are shown with the corresponding color bars in each panel. Unit: °C.

## Discussion

In this work, the results predict that clinical tSCS protocols may induce temperature rise of up to 9.4 °C in the skin layers which will be even larger for subjects with thicker SC or thinner dermis. The peak temperature magnitude and temperature spatial distribution depend on a combination of individual anatomical properties, stimulation configurations, and electrode sizes. We therefore recommend paying special attention to the individuals’ tissue thickness and blood perfusion properties when choosing proper stimulation protocols and alternatively taking measures to accelerate heat dissipation during tSCS clinical experiments. Our simulations with various anatomical models and stimulation properties consistently show that temperature rises are mainly distributed in the skin, fat, and abdomen, whereas the temperature variance of the CSF and WM/GM remains small and stable for most of the variables considered in this work except for the blood perfusion of the WM/GM. However, whether this change in thermal status could contribute to the neuromodulation of the neural activity deserves further study by referring to the thermal neuromodulation of infrared light (Wells et al., 2007; Peterson & Tyler, 2013) or microwave (Reverter et al., 2014).

Our results suggest that smaller-sized electrodes lead to higher injected current density and cause larger temperature rises. Similarly, in non-invasive transcranial direct current stimulation (tDCS) therapy, temperature rises were negligible with the conventional 5 × 7 cm rectangular electrode, whereas the temperature rise could be 0.55 °C in the brain tissues for the 4 × 1 ring electrode configuration with an electrode diameter approximately 1.1 cm (Datta, Elwassif & Bikson, 2009). Though small-sized electrodes may induce thermal damage, it is of great significance in neuromodulation. In clinical applications, proper electrode size should be chosen in accordance with the anatomical size of the subject’s and therapy’s requirement. In particular, in high-definition tSCS, small-sized electrode arrays are necessary to achieve a better stimulation focality in the non-invasive stimulation therapies (Nitsche et al., 2007; Dmochowski et al., 2011; Faria, Hallett & Miranda, 2011; Sadleir et al., 2012). A trade-off should be considered between the thermal issue and the stimulation accuracy before setting the clinical trials.

This work shows the findings that the temperature rise increases with stimulation intensity, consistent with previous work concerning the non-invasive tDCS bioheat transfer model (Datta, Elwassif & Bikson, 2009). Equation (2) indicates how the equivalent stimulation intensity was computed in this work, which is a non-linear form of the detailed stimulation parameters, such as the pulse width, pulse number, repeated frequency, and the peak intensity. From a biothermal safety standpoint, the commonly used biphasic stimulation waveforms may be disadvantageous despite being more efficient based on the balanced charge delivery criterion (Elwassif et al., 2006). This is due to the fact that more joule heat was generated by the larger equivalent intensity compared with monophasic stimulations. On the other side, in realistic stimulations, between every two pulses of the monophasic stimulation and during every stimulation cycle of both monophasic and biphasic stimulations, tissues in the stimulation electrical field have a period where they can cool, which may slow the temperature rise and delay the plateau. A better simulation method that enables monitoring of the electrical and thermal status of the long-term pulsed tSCS with acceptable computational consumption is necessary to investigate the temperature variance during the stimulation-off period and its impact on the plateau.

It is worth mentioning that the bioheat model used in this work is based on the classic Pennes equation. Although it has been widely used and proven to be valid, multiple new models were proposed in order to overcome its limitations (Charny, 1992), by considering the blood velocity field (Klinger, 1974; Wulff, 1974), dispersion and microcirculatory perfusion (Jiji, Weinbaum & Lemons, 1984), thermoregulation (Zolfaghari & Maerefat, 2010), or the temperature-dependent variability in tissue perfusion (Davies, Saidel & Harasaki, 1997; Lakhssassi, Kengne & Semmaoui, 2010). According to the simulation results of this work, in future experimental verifications, the time-dependent blood perfusion rate and sophisticated biological effects in the neural tissues should be considered as with the equation-unrelated factors concluded by Eugene’s work (Wissler, 2012). Moreover, as mentioned in “Effects of Blood Perfusion on the Temperature Distribution Induced by tSCS,” tissue burning is dependent on both the level of heating and exposure time. The degree of burning is predicted by calculating the fraction of necrotic tissue basing on the damage function as expressed by the Arrhenius equation (Henriques, 1947; Jiang et al., 2002). It indicates that the first, second, and third tissue burn occurs separately when the fraction of necrotic tissue reaches 0.411, 0.632, and 1, respectively. Future work might combine the Arrhenius model with more sophisticated bioheat model to evaluate the exact thermal damage caused by tSCS.

Note that the model used in this work is synthetic, consisting of 11 tissue types, which is different from reality. Actually, geometric irregularity of the spinal cord, especially the complex structure of the Vert and neural fibers through the horns, would affect the path of the electric field, which, in consequence, would influence temperature distribution. Moreover, other organs such as the kidney, liver and the intestine may affect the current path through the abdomen. This highlights the need for a more realistic biological model in future computational tSCS studies. Furthermore, based on the results of this work, the temperature rises during tSCS was mainly focused in the skin and fat layers which are tissues near the electrodes. In contrast, the deep tissues are protected from thermal damages due to the sparse effect and indirect contact with the electric sources. It is the skin’s structure that plays a significant role in determining the overall thermal status of the biological model. This conclusion inspires our future direction to work on a more detailed model of the skin similar to that of Gomez-Tames et al. (2016), to obtain more accurate and reliable predicted results.

## Conclusion

In this work, we built a human spinal cord model for a bioheat analysis in tSCS, in which the rise and spatial distribution of tSCS-induced temperature changes were monitored for 11 tissue types. Multiple factors that are thought to have an effect, including tissue thickness, blood perfusion rate, stimulation intensity, and electrode size, were quantitatively investigated. Systematic simulations and analysis of this work on the bioheat transfer could provide guidance for future tSCS applications in terms of reducing risk of thermal injury.

## Supplemental Information

10.7717/peerj.4921/supp-1 Supplemental Information 1 Parameters used in the simulations.

10.7717/peerj.4921/supp-2 Supplemental Information 2 Matlab codes of the simulation files used in this work.

10.7717/peerj.4921/supp-3 Supplemental Information 3 Raw data about the temperature of the biological tissues under different simulation conditions.

10.7717/peerj.4921/supp-4 Supplemental Information 4 Model files used in this work.

## Additional Information and Declarations

### Data Availability

The following information was supplied regarding data availability: The raw data are provided in the Supplemental Files.
